The article "Predictive Mathematical Models of the Short-Term and Long-Term Growth of the COVID-19 Pandemic" was published in 2021. Journal: Comput Math Methods Med.

# Predictive Mathematical Models of the Short-Term and Long-Term Growth of the COVID-19 Pandemic

**DOI:** 10.1155/2021/5556433

**Published:** 2021-08-11

**Authors:** Juan Luis Fernández-Martínez, Zulima Fernández-Muñiz, Ana Cernea, Andrzej Kloczkowski

**Affiliations:** ^1^Group of Inverse Problems, Optimization and Machine Learning, Department of Mathematics, University of Oviedo, Spain; ^2^Battelle Center for Mathematical Medicine, Nationwide Children's Hospital, Columbus, OH 43205, USA; ^3^Department of Pediatrics, The Ohio State University College of Medicine, Columbus, OH 43205, USA

## Abstract

The prediction of the dynamics of the COVID-19 outbreak and the corresponding needs of the health care system (COVID-19 patients' admissions, the number of critically ill patients, need for intensive care units, etc.) is based on the combination of a limited growth model (Verhulst model) and a short-term predictive model that allows predictions to be made for the following day. In both cases, the uncertainty analysis of the prediction is performed, i.e., the set of equivalent models that adjust the historical data with the same accuracy. This set of models provides the posterior distribution of the parameters of the predictive model that adjusts the historical series. It can be extrapolated to the same analyzed time series (*e.g.*, the number of infected individuals per day) or to another time series of interest to which it is correlated and used, *e.g.*, to predict the number of patients admitted to urgent care units, the number of critically ill patients, or the total number of admissions, which are directly related to health needs. These models can be regionalized, that is, the predictions can be made at the local level if data are disaggregated. We show that the Verhulst and the Gompertz models provide similar results and can be also used to monitor and predict new outbreaks. However, the Verhulst model seems to be easier to interpret and to use.

## 1. Introduction

An epidemic is the appearance of a particular disease in a large number of people at the same time and its corresponding spreading from person to person in a place where the disease is not permanently prevalent. When an epidemic has spread across the continents over the entire world it becomes a pandemic, a disease is called an endemic if it persists in a population. In the history of mankind, various pandemics have happened, some of which appear recurrently and others such as malaria, typhus, cholera, and sleeping sickness are endemic to some parts of the world (Snow [1]; Budd [2]).

Epidemiological models are designed to follow the dynamic of a disease transmission and study how it is spread and is being controlled in groups of people. Classical epidemic modeling was built on ordinary differential equations, the so-called population growth models. These models assume that the population is perfectly mixed, with people moving from the susceptible group, to the infected one, to the recovered (or dead) one. Within these groups, everyone is identical.

The article "Predictive Mathematical Models of the Short-Term and Long-Term Growth of the COVID-19 Pandemic" was published in 2021. Journal: Comput Math Methods Med.

The work of Bernoulli [3] concerning smallpox can be considered the first model in mathematical epidemiology. It was in the early 20th century, between 1900 and 1935, that the foundations of epidemiology were laid based on compartmentalized models (Ross [4]; Hamer [5]; Kermack and McKendrick [6]). Kermack and McKendrick's model considered a fixed population with three compartments, formed by the group of people who were likely to be infected at time *t*, *S*(*t*), the group of people who were infected, *I*(*t*), people who were able to spread the disease, and, *R*(*t*), the group of people who were not in the previous two groups, either because they had been immunized or because they had died as a result of the epidemic. This model is typically known under the acronym SIR. In its simplest formulation, it is applied to diseases with lifelong immunity, i.e., once recovered patients cannot be susceptible again. In this model, births and deaths are not taken into account because the duration of the disease is too short compared to the life of an individual, so that the total population, *N*, is considered constant. Representing by *S*(*t*),  *I*(*t*), and *R*(*t*), the number of susceptible, infected, and recovered individuals, we have the following: *N* = *S*(*t*) + *I*(*t*) + *R*(*t*), where *N* is the total population.

The SIR model can be written as follows:

(1) $$\begin{array}{c} \left\{\begin{array}{c} \frac{dS\left(t\right)}{dt}=-\frac{r\;S\left(t\right)I\left(t\right)}{\text{N}},\\ \frac{dI\left(t\right)}{dt}=\frac{r\;S\left(t\right)I\left(t\right)}{\text{N}}-cI\left(t\right),\\ \frac{dR\left(t\right)}{dt}=cI\left(t\right), \end{array}\right. \end{array}$$

where *r* is the infectious rate or the probability of transmitting disease between a susceptible and an infectious individual and *c* is the recovery rate determined by the average duration of infection.

The values of parameters *r* and *c* should be estimated and adjusted so that they can justify the excess of deaths.

A modification of the SIR model consists in conflict considering births and deaths rates (*μ* and *α*, respectively):

(2) $$\begin{array}{c} \left\{\begin{array}{c} \frac{dS\left(t\right)}{dt}=\text{N}-\frac{b\;S\left(t\right)I\left(t\right)}{\text{N}}-S\left(t\right),\\ \frac{dI\left(t\right)}{dt}=\frac{b\;S\left(t\right)I\left(t\right)}{\text{N}}-cI\left(t\right)-I\left(t\right),\\ \frac{dR\left(t\right)}{dt}=cI\left(t\right)-R\left(t\right). \end{array}\right. \end{array}$$

A variant of the SIR model is the SEIR [7], which considers an incubation period during which individuals have been infected but are not yet infectious themselves, with *E*(*t*) being the exposed group. The SEIS variant is like SEIR, but in the end, the immunity is not acquired. If there is a passive immunity and a latency period, we have the MSEIR model and if the R-class immunity is temporary and individuals in this group may become susceptible again, then we have the MSEIRS model (see Brauer [8] for more details about models for pandemics). Many scientists have chosen to use the SIR model (Bärwolff [9]; Weiss [10]) or one of its variants (Peng et al. [11]; Tian et al. [12]; Tsay et al. [13]; Prem et al. [14]; Hethcote [15]) and even have designed some improved variants applicable to COVID-19 that take into account, among other things, undetected infectious cases (Ivorra et al. [16]) or time-delay (Shao et al. [17]).

The article "Predictive Mathematical Models of the Short-Term and Long-Term Growth of the COVID-19 Pandemic" was published in 2021. Journal: Comput Math Methods Med.

All these prediction models, although they have different levels of complexity, follow the first phase of adjustment, where an inverse problem to identify their critical parameters is solved. In this phase, the values of the model parameters that constitute the model are being adjusted to the historical data with a minimum mismatch, that is, the epidemiological model is able to reliably predict the past. Once these parameters have been obtained, the model is used to predict the evolution of the disease in the future. One of the limitations of these SIR-type models is having at disposal the population *R*(*t*) to identify the parameters.

In SIR-type models, a fundamental parameter is the basic reproduction number *R*₀ which measures the average number of people infected by each sick person. As can be expected, this number differs greatly and depends on the social behavior of the given population, since living in isolation in rural areas is completely different than living in large cities, where it is difficult to maintain the social distance. For that reason, some authors have stated that the variation range for this parameter is 2 to 2.6 (Ferguson et al. [18]; Massonnaud et al. [19]; Li et al. [20]). Other authors estimate this interval to be between 1.5 and 3 (Massonnaud et al. [19]) or even greater than 5 (Sanche et al. [21]), depending on the areas of study. As we will see in this paper, this great variation might be related not only to the epidemiological problem itself but also to the uncertainty space of this parameter in the inverse problem. All these models need a good quality data from the several compartments into which the collected data is being divided.

The article "Predictive Mathematical Models of the Short-Term and Long-Term Growth of the COVID-19 Pandemic" was published in 2021. Journal: Comput Math Methods Med.

A different and simpler approach to model pandemics consists of treating the outbreak as a population growth model. In this case, the model is applied to the infected people. Particularly, the limited growth models, such as the logistic one proposed by Verhulst [22], might be used to understand and predict the pandemics. This population model takes into account that competition between individuals for a limited resource leads to a limited growth. The time before the population reaches half of its limit value (or maximum capacity) is the period of rapid growth. After, the growth rate decreases to reach zero in a period of reduced growth to stabilize the total number of individuals of the population to its maximum value. The logistic model has been used to study the evolution of COVID-19 by different authors (Dattoli et al. [23]; Zeng et al. [24]; Cherniha and Davydovych [25]; Cakir and Savas [26]).

Another interesting model used in biology for the growth analysis is the Gompertz model (Gompertz [27]), which has been used to describe the growth of animals and plants and also the volume of bacteria and cancer cells ([28]; Tjørve and Tjørve [29]).

Although the underlying law is different from the Verhulst model, the conclusions that might be achieved to predict the evolution of a population might be similar if the prediction is correctly performed. This paper is aimed to show that the COVID-19 outbreak can be modeled via the Verhulst population model to predict the evolution of the disease with the aim of planning of the demand for the health care resources and to minimize deaths by adopting the right decisions. Besides, a short-term prediction of the medical needs can be utilized to predict the hospital bed admissions and the urgent care needs. The long-term forecasts could be used to estimate when the peak of the pandemic will be reached and to monitor the probability of a new outbreak. To perform these tasks properly, the inverse problems of the Verhulst forward model should be analyzed with its corresponding uncertainty analysis.

The Verhulst model depends only on three parameters that should be identified based on historical data: the initial population of the infected individuals, the rate of growth that is constant and serves to explain globally the expansion of the outbreak, and the maximum number of people who will be infected. The uncertainty space of the Verhulst model is composed of a set of three-dimensional parameters that fit the historical data within the same error bounds. These models are called equivalent and they are located on curvilinear valleys of the cost function topography map (Fernández Martínez et al. [30]). The uncertainty in inverse problems is due to the noise in data and due to modeling assumptions, that is, the existing tradeoff among parameters. The sampling of this set of equivalent models serves to quantify the uncertainty in the past and to translate it to the future prediction by providing the percentile curves of the outbreak. These percentile curves make the methodology of predicting the outbreak more robust for public health purposes, since the observed data of the outbreak fits to one percentile curve along with the history. The median curve (or percentile 50) is the most likely. Therefore, if the outbreak goes below the median curve, it is under control. Conversely, if the outbreak goes below the percentile 75-90, the outbreak is uncontrolled, and a future growth of infections has to be expected. We show the application to the outbreak prediction worldwide and other examples. We have shown that the Verhulst and the Gompertz models provide similar results and both can be also used to monitor and predict new outbreaks, with the Verhulst model being easier to interpret and to use. Additionally, we have performed the uncertainty analysis of the predictions, by constructing the set of equivalent models that adjust the historical data with the same accuracy, and could be extrapolated to predict the number of patients admitted to urgent care units, the number of critically ill patients, or the total number of admissions. Such predictions are extremely important for medical authorities for prevention planning during a pandemic.

The article "Predictive Mathematical Models of the Short-Term and Long-Term Growth of the COVID-19 Pandemic" was published in 2021. Journal: Comput Math Methods Med.

## 2. Methodology

### 2.1. Long-Term Forecasting via Verhulst Model

The Verhulst model is a limited-growth population model, which assumes that population growth is limited by population size, fertility, and the amount of available resources. This causes that the population converges towards a stationary solution. The Verhulst model is a modification of the Malthus model (1766-1834) that predicted the exponential growth of the population. The Verhulst model corresponds to the first-order differential equation:

(3) $$\begin{array}{c} \frac{dP}{dt}=rP\left(1-\frac{P}{K}\right),\\ P\left(0\right)=P_{0}, \end{array}$$

where *P*(*t*) is the population size, which depends on time, *r* is the growth rate (or decline), and *K* is the carrying capacity of the medium and represents the maximum number of individuals that the population can support. In our case, it is the maximum number of people that is going to be infected by the virus.

The growth rate gr (*t*) is in this case:

(4) $$\begin{array}{c} \text{gr }\left(t\right)=\frac{dP\left(t\right)/dt}{P\left(t\right)}=r\left(1-\frac{P\left(t\right)}{K}\right), \end{array}$$

which is not constant but self-regulates according to the term (1 − *P*(*t*)/*K*) which takes into account the distance between the size of the population at any given time *P*(*t*) and the maximum capacity (*K*). Besides, when *P*(*t*) approaches *K*, gr (*t*) goes to 0. This is the main difference to the well-known Malthus model, where gr (*t*) = *r* ∈ ℝ. The general solution of the Verhulst model is

(5) $$\begin{array}{c} P\left(t;A\right)=\frac{K}{1+Ae^{-rt}}, \end{array}$$

where *A* is a real constant that has to fulfill the initial condition *P*(0) = *P*_0_

(6) $$\begin{array}{c} P_{0}=\frac{K}{1+A}. \end{array}$$

Therefore, we have

(7) $$\begin{array}{c} P\left(t\right)=\frac{KP_{0}e^{rt}}{K+P_{0}\left(e^{rt}-1\right)}. \end{array}$$

The Verhulst model can adequately represent the spread of an epidemic at the beginning, when the epidemic spreads rapidly, as each infected person is susceptible to infect other individuals. As the number of infected people grows, it is more and more difficult to find a person who has not been previously in contact with the disease. This is the reason for the limited growth, independently to the imposed lockdowns.

The article "Predictive Mathematical Models of the Short-Term and Long-Term Growth of the COVID-19 Pandemic" was published in 2021. Journal: Comput Math Methods Med.

Equation (5) provides the total number of infected individuals in time *t*, while Equation (1) provides the number of newly infected people per day, i.e., the speed of infection. The *P*(*t*) curve is sigmoidal in shape and is called the logistic curve, while the (*dP*(*t*))/*dt* curve is bell-shaped and reaches its maximum in time *t*_max_:*P*(*t*_max_ ) = *K*/2, that is, when the total number of infected people reaches the half of population. The maximum of *dP*(*t*)/*dt* at *t*_max_ is

(8) $$\begin{array}{c} \max{\left(\frac{dP\left(t\right)}{dt}\right)}_{t=t_{\max}}=\frac{rK}{4}. \end{array}$$

At that point, the *P*(*t*) curve has a tipping point, so the growth rate of the pandemic goes from increasing to decreasing values. This model has the advantage of being simple, robust, and easy to understand.

Equation (8) is very useful to determine the maximum total number of people infected from the maximum daily number of people infected, knowing the rate of growth *r*.

Also, it is very easy to model the effect of the vaccines, considering a factor *α* of immunity in the population. The effect is similar to considering the growth rate being *r*(1 − *α*) after vaccination. This is obviously a model. For instance, if *r* = 0.15 and *α* = 0.3 (30% of the population is immune), then, the rate will decrease to *r*(1 − *α*) = 0.105.

### 2.2. The Gompertz Model

Another model that can be used to fit the total number of infected persons is the Gompertz model

(9) $$\begin{array}{c} \frac{dP}{dt}=rP\ln\left(\frac{K}{P}\right),\\ P\left(0\right)=P_{0}. \end{array}$$

Its general solution is

(10) $$\begin{array}{c} P\left(t\right)=Ke^{-Be^{-rt}}, \end{array}$$

where *K* describes the maximum infected population, *B* is a real constant that establishes the movement of the curve along the *x*-axis, and *r* is the growth rate. All these parameters are positive. In this case, the growth rate gr (*t*) is logarithmic:

(11) $$\begin{array}{c} \text{gr }\left(t\right)=\frac{dP\left(t\right)/dt}{P\left(t\right)}=r\ln\left(\frac{K}{P}\right). \end{array}$$

Since *P*(0) = *Ke*^−*B*^, *K* can be expressed as a function of *P*(0); therefore, we have

(12) $$\begin{array}{c} P\left(t;P_{0},B,r\right)=P_{0}e^{-B\left(e^{-rt}-1\right)}, \end{array}$$

that depends on three parameters, *P*_0_, *B*, and *r*. The number of new infected is given by *dP*(*t*)/*dt*. However, we see in the real practice that due to the existing trade-offs, parameters of the Gompertz model are more difficult to identify.

The article "Predictive Mathematical Models of the Short-Term and Long-Term Growth of the COVID-19 Pandemic" was published in 2021. Journal: Comput Math Methods Med.

The time when the total number of infected individuals reaches the half of the population occurs when 1/2 = *e*^−*Be*^−*rt*^^, that is, *t*_*K*/2_ = −ln(ln(2/*B*))/*r*. Besides, the maximum increase occurs at *t*_max_ = ln(*B*)/*r*, and the increase at *t*_max_ is

(13) $$\begin{array}{c} \max{\left(\frac{dP\left(t\right)}{dt}\right)}_{t=t_{\max}}=\frac{Kr}{e}>\frac{Kr}{4}, \end{array}$$

which is higher than the one corresponding to the Verhulst model (*Kr*/4). Therefore, for the same values of *K* and *r*, the maximum increase of the Gompertz curve is bigger than for the Verhulst model.

In both cases, the inverse problem has three similar parameters to be identified, namely, *K*, *P*_0_, and *r*.

In the case of the Gompertz model, the natural parameters to be identified are *B*, *P*_0_ and *r*. The following relationship

(14) $$\begin{array}{c} \ln K=\ln P_{0}+B, \end{array}$$

relates *B* and *P*_0_ with the maximum number of infected people, *K*.

Besides, gr (*t*) = *rBe*^−*rt*^. Therefore,

(15) $$\begin{array}{c} \ln\left|\frac{dP\left(t\right)/dt}{P\left(t\right)}\right|=\ln\left(rB\right)-rt. \end{array}$$

This last expression can be used to obtain a first approximation of *r* and *B* by a linear regression. A different possibility consists in taking logarithms in Eq. (10)

(16) $$\begin{array}{c} \ln P\left(t\right)=\ln P_{0}-B\left(e^{-rt}-1\right), \end{array}$$

and solving Eq. (16) iteratively as follows:

1. Considering an initial guess for *r* = 0.1
2. Identifying *P*_0_ and *B* by solving the linear system (Eq. (16)) by least-squares, by writing (16) for different times *t*_*k*_
3. Identifying *r* by solving -ln|(ln(*P*_0_/*P*(*t*))/*B*) + 1| = *rt* by scalar least-squares, using the same approach mentioned in step 2
4. The iterative procedure stops when ‖**P** − **P**^∗^‖_2_ is smaller than a given bound

The article "Predictive Mathematical Models of the Short-Term and Long-Term Growth of the COVID-19 Pandemic" was published in 2021. Journal: Comput Math Methods Med.

## 3. The Prediction Problem and the Inverse Problem

The Verhulst model and the Gompertz model depend only on three parameters to be identified:

- The initial population of infected persons (*P*_0_) who spread the virus. Its default value is 1, but it must be correctly identified since it may not coincide with the number of infected people detected on the first day when the statistics were initiated
- The intrinsic growth rate (*r*). This parameter provides a global overview of the outbreak
- The maximum population or load capacity, *K*

Knowing (identifying) these three parameters, it is relatively simple to simulate the growth of the outbreak.

In this case, the theoretical model considers that the daily number of infected people at time *t*, *dP*(*t*)/*dt*, can be described as a temporal stochastic process:

(17) $$\begin{array}{c} \frac{dP\left(t\right)}{dt}=\mu \left(t\right)+R\left(t\right), \end{array}$$

where *μ*(*t*) is the deterministic trend and *R*(*t*) is the stochastic unpredictable residual, which has no temporal correlation structure. Besides, the trend *μ*(*t*) is supposed to follow any of the two models (Verhulst/Gompertz), which is *dP*(*t*)/*dt* ≈ *μ*(*t*). Therefore, the Verhulst and the Gompertz models can only explain the trend *μ*(*t*) of *dP*(*t*)/*dt*, and the difference between both are high-frequency increments that are due to the local time behavior of the pandemic. It is important to understand that the low-frequency part of model, *μ*(*t*), and the high-frequency content, *R*(*t*), have different uncertainty spaces. In fact, the Verhulst/Gompertz deterministic models are only able to mimic *μ*(*t*), while the term *R*(*t*) has almost no temporal correlation and should be modeled as white noise. The white noise can be Gaussian white if the noise values are mutually uncorrelated with zero mean and have the same Gaussian probability distribution. In time series analysis, there are often no explanatory variables other than the past values of the variable being modeled. In this case, the noise process can be modeled as a moving average process, in which the current value of the dependent variable depends on the current and past values of a sequential white noise process.

Figure 1 shows the dynamics of the pandemic for three different cases with maximum populations of 500 000, 800 000, and 1 million people and intrinsic growth rates of 0.1 and 0.2.

It can be observed that the peak of the curve of new infections has a maximum at the inflection point of the curve of total infections, so its temporal location is very well determined. Besides, as it was detailed, it corresponds to the time in which half of the maximum population is reached. Another remarkable circumstance is that the support of the curve of new infected varies in this case between 60 and 75 days, which would be the characteristic time necessary for it to be controlled.

The article "Predictive Mathematical Models of the Short-Term and Long-Term Growth of the COVID-19 Pandemic" was published in 2021. Journal: Comput Math Methods Med.

Figure 2 shows the same simulations using the Gompertz model with the same parameters as for the Verhulst model. In this case, the disappearance of the pandemic is faster. This fact indicates that the growth parameter for the Gompertz model should be smaller to be compared to the results of the Verhulst model.

Please note that both predictions shown in Figures 1 and 2 are smooth and do not contain high-frequency variabilities observed in the real data.

The inverse problem can be written as follows: given a time series of the total number of people infected till time *t*_*n*_: {(*t*_1_, *P*_1_), (*t*_2_, *P*_2_), ⋯., (*t*_*n*_, *P*_*n*_)}  finding the set (or sets) of parameters **m** = (*K*, *P*_0_, *r*) such that the observed data  **d**^**obs**^ = (*P*_1_, *P*_2_, ⋯, *P*_*n*_) ∈ ℝ^*n*^ is fitted with an error smaller than a given error bound: *tol*.

Calling **F**(**m**) to the forward prediction model (the Verhulst/Gompertz growth model in this case), it is, to sample the uncertainty space of this inverse three-dimensional problem:

(18) $$\begin{array}{c} M_{tol}=\left\{m=\left(K,P_{0},r\right)\text{: }\frac{{\left\|F\left(m\right)-d^{obs}\right\|}_{1}}{{\left\|d^{obs}\right\|}_{1}}\leq tol\right\}. \end{array}$$

Equation (8) holds for any norm to measure the relative data misfit ‖**F**(**m**) − **d**^**obs**^‖_1_/‖**d**^**obs**^‖_1_. In this case, the *L*_1_ norm has been adapted because of its robustness to the presence of outliers. The aim of this analysis is to identify the set of models **m** = (*K*, *P*_0_, *r*) that fits the historical data with a similar precision. This procedure takes into account the topography of the cost function in nonlinear inverse problems (Fernández-Martínez et al. [30, 31]) and the effect of noise on the observed data (Fernández-Martínez et al. [32, 33]) which deforms this topography and falsifies the identification of the best model. Besides, it has been shown (Fernández-Martínez et al. [30, 31]) that the so-called equivalent models belong to flat curvilinear valleys of the objective function in which the latter reaches similar values. These models can be also located in different disconnected basins of the cost function landscape. In the case of linear inverse problems, this uncertainty region is unique (bounded or not). The uncertainty analysis consists of obtaining a representative sample of these models through sampling or global optimization techniques (Fernández-Martínez [34]). In that sense, the technique consisting of finding the model with the maximum plausibility (with the least fitting error of the historical data) is inadequate since no different scenarios are contemplated. In addition, the technique of providing prediction confidence intervals is mostly based on the hypothesis of linearity (normality). This hypothesis is not needed in this approach since the posterior distribution of the prediction is in this case given. It should be noted that the prediction percentile curves have a much more complex shape than that anticipated by a single (most accurate) predictive model, regardless of its type (SIR, Verhulst, etc.). The reason is that percentile curves collect the contribution of different plausible scenarios, not only the one with the smallest historical fitting error.

The article "Predictive Mathematical Models of the Short-Term and Long-Term Growth of the COVID-19 Pandemic" was published in 2021. Journal: Comput Math Methods Med.

Other global optimization methods such as genetic algorithms or simulated annealing could be used to solve this low-dimensional inverse problem. Nevertheless, the most important feature is the capability of performing a good sampling of the posterior distribution of the model parameters. With PSO, the sampling during the optimization can be done much faster than with other methods, as shown by Fernández Alvarez et al. [35] and Fernández Martínez et al. [36] who compared these various algorithms.

Once this set of equivalent models have been sampled, it is possible to extrapolate the pandemic curve *ad-futurum* by taking into account all these sampled models that fit the historical data equally well and to determine the different percentiles of the posterior distribution of the number of infected during the outbreak (daily ones and cumulated). That way, the uncertainty in the future prediction is implemented.

Numerical data can be sorted in increasing or decreasing order by setting a rank order. A percentile is a value at a particular rank. The *p*-percentile of the *ad-futurum* prediction on day *t* is the number of infected people left by the *p*% of predictions below. The 10^th^, 25^th^, 50^th^, 75^th^, and 90^th^ percentiles are determined. The percentiles curves for Verhulst and Gompertz models are generated by applying this concept to the set of predictions in each time, that is, calling (*I*_1_^∗^, *I*_2_^∗^, ⋯, *I*_*q*_^∗^) ∈ ℝ^*q*^ the set of predictions in time *t*_*k*_, the percentile *p* is *I*_*p*_: *P*(*I*_*k*_^∗^ < *I*_*p*_). This probability is inferred from the set of equivalent predictions (*I*_1_^∗^, *I*_2_^∗^, ⋯, *I*_*q*_^∗^).

The article "Predictive Mathematical Models of the Short-Term and Long-Term Growth of the COVID-19 Pandemic" was published in 2021. Journal: Comput Math Methods Med.

That way, the reality (the number of infected observed cases) on that same day (once predicted before) is an additional curve of the model. The 50^th^ percentile or median is the most likely value of the predicted values, since it is the center of the posterior distribution. If the evolution of the pandemic goes towards lower percentiles (below the median), then the pandemic would be under control. Conversely, if the pandemic evolves towards higher percentiles, then the opposite can be concluded. This methodology is consistent with the Bayesian approach to inverse problems (see for instance Tarantola [37]) consisting in sampling the posterior distribution of the model parameters in inverse problems to adopt risk decisions. This methodology is commonly adopted in many fields of the technology.

One of the questions that is always discussed is to which degree the pandemic (number of infections) could be extrapolated in time. For that purpose, we can use the correlogram which takes into account the memory of the temporal series.  Figure 3 shows the absolute variogram and the stationary covariance of the daily infected in Spain. It can be observed that the variogram reaches a plateau between 40 and 60 days, and the covariance cancels out in 138 days. Therefore, the correlation memory is at least longer than one month. Thus, it is completely licit to perform *ad-futurum* predictions of the trend that long.

Although not shown in the paper, the correlation of the term *R*(*t*) after filtering out the trend is lower than 2 days, which coincides with the observed delay in the data variability provided by the Spanish authorities. This fact means that *R*(*t*) could be modeled as a white noise.

## 4. RR-PSO Sampling

The sampling of the equivalent model parameters in (8) that fit the historical data is done via global optimization. The sampling is performed with the Regressive-Regressive Particle Swarm Optimization (RR-PSO) algorithm (Fernández Martínez and García-Gonzalo [38]) which is a member of the Particle Swarm Optimization (PSO) family. The PSO algorithm (Kennedy and Eberhart [39]) is a global optimization algorithm that was initially bioinspired by the bee swarms foraging for food. The bees, when foraging for pollen, explore the region where there is the highest density of flowers so that the probability of finding pollen is higher. PSO uses a swarm of models **m** (called particles) to explore an *n*-dimensional space of plausible solutions in order to optimize the data prediction error. Initially, a swarm of model parameters is randomly initialized within the search space. These are the only constraints or piece of prior information that it is needed for the PSO algorithm to work. As PSO progresses, the positions of the model parameters in the search space are updated as follows:

(19) $$\begin{array}{c} \begin{array}{c} v_{\text{i}}^{\text{k}+1}={\omega v}_{\text{i}}^{\text{k}}+\emptyset_{1}\left(g^{\text{k}}-x_{\text{i}}^{\text{k}}\right)+\emptyset_{2}\left(l_{\text{i}}^{\text{k}}-x_{\text{i}}^{\text{k}}\right),\\ x_{\text{i}}^{\text{k}+1}=x_{\text{i}}^{\text{k}}+v_{\text{i}}^{\text{k}+1}. \end{array} \end{array}$$

Here, **x**_i_^k^ is the *i*th model in the *k*th iteration, and **v**_**i**_^**k**^ its velocity, that is, the model perturbations needed to minimize the cost function. The velocity update depends on **l**_**i**_^**k**^  which is the *i*th particle's best position, and on **g**^k^, which is the global best position among all **l**_**i**_^**k**^ positions. Mathematically is a double stochastic gradient algorithm in the model space. The PSO parameters, ∅_1_ = r_1_a_g_ and ∅_2_ = r_2_a_l_, are the random global and local accelerations, and *ω* is a real constant called inertia weight, while *r*_1_ and *r*_2_ are uniform random variables in the interval [0, 1], used to weight the global and local acceleration constants *a*_*g*_ and *a*_*l*_. These are three PSO tuning parameters needed to achieve stability of the PSO particle trajectories (Fernández Martínez and García Gonzalo [40]) and to explore of the cost function landscape.

The article "Predictive Mathematical Models of the Short-Term and Long-Term Growth of the COVID-19 Pandemic" was published in 2021. Journal: Comput Math Methods Med.

From the physical point of view, PSO can be interpreted as a double stochastic gradient algorithm in the model space and is the particular case of the generalized PSO (GPSO) algorithm (Fernández Martínez and García Gonzalo [41]) for *t* = *k* and a unit time-step (∆*t* = 1):

(20) $$\begin{array}{c} \begin{array}{c} v_{i}\left(t+∆t\right)=v_{i}\left(t\right)\left[1-\left(1-\omega \right)∆t\right]+\emptyset_{1}∆t\left[g\left(t\right)-x_{i}\left(t\right)\right]\;+\emptyset_{2}∆t\left[l_{i}\left(t\right)-x_{i}\left(t\right)\right],\\ x_{i}\left(t+∆t\right)=x_{i}\left(t\right)+v_{i}\left(t\right)\left(t+∆t\right)∆t. \end{array} \end{array}$$

This and other models of the PSO family were obtained from the PSO continuous model (Fernández Martínez and García Gonzalo [41]) which is a stochastic damped mass-spring system. In this paper, we have used the Regressive-Regressive PSO (RR-PSO) which is a member of the PSO family that was obtained from the PSO continuous model by adopting regressive discretization in acceleration and in velocity (Fernández Martínez and García-Gonzalo [38]). RR-PSO can be written as follows:

(21) $$\begin{array}{c} \left\{\begin{array}{c} v_{i}\left(t+∆t\right)=\frac{v_{i}\left(t\right)+\emptyset_{1}∆t\left[g\left(t\right)-x_{i}\left(t\right)\right]+\emptyset_{2}∆t\left[l_{i}\left(t\right)-x_{i}\left(t\right)\right]}{1+\left(1-\omega \right)∆t+\emptyset ∆t^{2}},\\ x_{i}\left(t+∆t\right)=x_{i}\left(t\right)+v_{i}\left(t+∆t\right)∆t,\\ x_{i}\left(0\right)=x_{0},\\ v_{i}\left(0\right)=v_{0}, \end{array}\right. \end{array}$$

where (*t*, ∆*t*) ∈ ℝ.

The article "Predictive Mathematical Models of the Short-Term and Long-Term Growth of the COVID-19 Pandemic" was published in 2021. Journal: Comput Math Methods Med.

RR-PSO was chosen among the different members of the PSO family due to its optimum balance between the exploration and exploitation capabilities. This feature is very important for sampling the region of equivalent models. Besides, the tuning of the RR-PSO parameters is very simple since they are aligned in a straight line (Fernández Martínez and García-Gonzalo [38]). This type of global algorithms does not need prior information or regularization term to perform the optimization. They only need the design of the search space, which is a prism in this particular case in three dimensions.

In our case, the bees are the parameters of the Verhulst/Gompertz models, **m** = (*K*, *P*_0_, *r*), and the density of pollen is related to the value of the misfit obtained in fitting the historical data. In the case of the Verhulst model, the search space is automatically designed by solving the discrete difference equation:

(22) $$\begin{array}{c} P\left(t+1\right)-\left(1+r\right)P\left(t\right)+\frac{r}{K}P^{2}\left(t\right)=0,\\ P\left(0\right)=P_{0}. \end{array}$$

This differential equation can be written as

(23) $$\begin{array}{c} P\left(k+1\right)-P\left(k\right)=aP\left(k\right)+bP^{2}\left(k\right),k=1,\cdots ,s-1, \end{array}$$

where *s* is the number of data observed in the history of the outbreak.

It is straightforward to identify through the least-squares the parameters *a*, *b*. Based on these values, it is straightforward to design the low and the upper search limits for *r* and *K*. In the case of *P*_0_, it is simpler since this parameter is usually better constrained. Given a set of particles **m** = (*K*, *P*_0_, *r*) in the search space, the cost function to be optimized is the distance in the *L*_1_ norm between the observed infected data and the data predicted with this model:

(24) $$\begin{array}{c} C\left(m\right)=\frac{{\left\|P^{\text{obs}}-P^{*}\left(m\right)\right\|}_{1}}{{\left\|P^{\text{obs}}\right\|}_{1}}100+C_{1}\left(m\right). \end{array}$$

Besides, in (24), a term including the fitting of the velocity is included, *C*_1_(**m**), to improve the fitting of the daily curve as well:

(25) $$\begin{array}{c} C_{1}\left(m\right)=\alpha \frac{{\left\|{dP}^{\text{obs}}-{dP}^{*}\left(m\right)\right\|}_{1}}{{\left\|{dP}^{\text{obs}}\right\|}_{1}}100, \end{array}$$

where **dP**^obs^, **dP**^∗^(**m**) are the observed and predicted daily increments, and *α* a real parameter used to specify the weight of the term *C*_1_(**m**).

The article "Predictive Mathematical Models of the Short-Term and Long-Term Growth of the COVID-19 Pandemic" was published in 2021. Journal: Comput Math Methods Med.

As specified in Eq. (18), in the posterior analysis, we will only choose the parameters that guarantee that the prediction error is lower than the admitted tolerance (error bound) that is tuned to take into account the high-frequency content of the outbreak, such as sudden infections in retirement homes or in social meetings that do not respect social distancing and the corresponding health protection measures.

The flowchart followed in this paper is as follows:

- Inverse modeling and the uncertainty analysis of the COVID-19 outbreak via the Verhulst/Gompertz models
- *Ad-futurum* prediction of the outbreak
- Cross-correlation of the number of infected temporal series with other time series (health needs)
- *Ad-futurum* prediction of the cross-correlated time series

## 5. Results

In this section, we show the application of this methodology to the COVID-19 outbreak in Spain.  Figure 4 shows the daily number of infected individuals in Spain from the beginning of the outbreak. It can be observed that the first wave of the pandemic begins around March 2020, and its intensity is lower due to the confinement. Also, the number of positive cases was undersampled because the tests were mostly performed only during hospital admissions. Then, we observe the second wave of the pandemic that begins in July and ends in December 2020. The third wave begins after Christmas 2020 due to the preholiday relaxing of the lockdown restrictions because of the social and economic pressures. The abovementioned population models can interpret every wave individually by shifting the time origin.

For instance, Figure 5 shows the analysis of the third wave in Spain. This figure shows the posteriori distribution of the predicted daily number of infected people computed on February 2, 2021. The beginning of the third wave was set on December 12, 2020. This figure shows the observed data, its temporal trend, and different percentiles curves (P10, P25, P50, P60, P75 P90, and P95) of the prediction. The percentiles curves were generated using the methodology that was previously explained, that is, performing the sampling of the equivalent models that fit the historical data and extrapolating these predictions *ad-futurum*. We also provide the trend that is calculated via the spectral filtering of the data series.

Our interpretation is that the outbreak achieved its maximum around January 21, 2021, when the daily infection maximum was located on the P90 curve. This situation also happened one week before, but the outbreak continued to increase after a brief period of decrease. This is interpreted as noise in data, mainly introduced by the weekends or some delays in the data analysis transfer. According to our prediction from the model, the third wave will be under control by the end of March 2021. The maximum number of the infected people seems to approach 2 million as seen in the P75 curve of the lower plot displaying the total number of infections.

The article "Predictive Mathematical Models of the Short-Term and Long-Term Growth of the COVID-19 Pandemic" was published in 2021. Journal: Comput Math Methods Med.

The percentile curves serve to detect the risk of new resurgence and monitoring new outbreaks. Assigning a risk of regrowth from the percentile curves is automatic:

- If the number of newly infected cases is less than P10: very low risk
- Between P10 and P25: low risk
- Between P25 and P50: low to medium risk
- Between P50 and P75: medium to high risk
- Between P75 and P90: high risk
- Above P90: very high risk—out of control

Figure 6 shows the histograms of *K* and *r* parameters identified by RR-PSO in predicting the number of infected people. The maximum number of infected individuals was 1.5 million people. The intrinsic growth rate of the infection is between 0.08 and 0.10. Obviously, this value depends on the type of society, its mobility, density of population, and the health conditions.

Also, one of the major questions in the modeling is to decide if the outbreak has achieved its maximum. The derivative of the number of daily infected cases is a very interesting tool to elucidate this question. The lower plot in Figure 7 shows the second derivative of *P*(*t*), that is calculated by numerical differentiation of the trend (*μ*(*t*)) of *dP*(*t*)/*dt*. The fact that the second derivative is close to zero indicates that we are close to a peak, but unfortunately, it is possible to have a local reversal in the trend.

### 5.1. Short-Term Prediction

Long-term forecasting can be complemented by short-term (next day) forecasting using a time series analysis method.  Figure 8 shows the application of such a method for the next-day prediction of the number of infected cases, the most likely value being the median. The interquartile range can also be determined, as well as the minimum and maximum percentiles that provide the one-day limits on the evolution of the pandemic. As it was already explained, above the 90th percentile provides a very high probability of a new out of control outbreak. This method of short-time prediction can also be used to predict health care needs (admissions, ICUs, critical care patients, deaths), by correlating the corresponding time series with the series numbers of infected people, and by transmitting the uncertainty of the prediction of new COVID-19 infections to these predictions. The method works as follows:

- Performing a linear regression between the health care needs (*H*) and the daily infected

(26) $$\begin{array}{c} H\left(I\right)=a_{1}I+a_{0}., \end{array}$$

(ii) Given a set of equivalent predictions of *I*, constructing the percentiles for *H*, taking into account (26).

The article "Predictive Mathematical Models of the Short-Term and Long-Term Growth of the COVID-19 Pandemic" was published in 2021. Journal: Comput Math Methods Med.

This allows for a much more effective control of the effects of the pandemic and an intelligent and automated forecast of hospital needs.

### 5.2. Prediction via the Gompertz Model

Finally, the same methodology could be employed with the Gompertz model.  Figure 9 shows the modeling of the third outbreak in Spain via the Gompertz model. Both the Verhulst and the Gompertz models provide similar answers. Nevertheless, the Gompertz model is more sensible to the initial population (due to Eq. (14)) than the Verhulst model whose parameters are simpler to tune.

## 6. Conclusions

This paper presents the Verhulst and the Gompertz models for predicting the effects of the COVID-19 outbreak and helping on decision-making, both in terms of health care needs and public health outcomes. These models depend only on three parameters (the initial number of infected individuals, the maximum number of infected people, and the infection growth rate), which can be identified by fitting the historical data. The uncertainty analysis of these prediction models serves to determine the posterior distribution of the predictions for the daily infections and to translate the effect of this uncertainty to the future, via the percentile curves. These models serve to perform long-term and short-term predictions that can be used to anticipate future health care needs and the arrival of a next wave of the pandemic. We show several examples for the COVID-19 prediction in Spain. Interestingly, the intrinsic growth rate of the infection is between 8% and 10%, which indicates that the SARS-CoV-2 virus effects on average 8 to 10 people for every 100 susceptible cases. It is expected that this number will decrease in the future due to the effect of mass vaccination. We also have shown that the Verhulst and the Gompertz models provide similar results; however, the parameters in the Verhulst model are easier to tune. In view of these circumstances, the use of the Verhulst model seems more appropriate and more intuitive than that of Gompertz.

## Figures and Tables

**Figure 1:** Simulation of the dynamics of a pandemic according to the Verhulst model for different values of load capacity and intrinsic growth rate.

**Figure 2:** Simulation of the dynamics of a pandemic according to the Gompertz model for different values of load capacity and intrinsic growth rate.

**Figure 3:** Absolute variogram and stationary covariance for the Spanish COVID-19 outbreak.

The article "Predictive Mathematical Models of the Short-Term and Long-Term Growth of the COVID-19 Pandemic" was published in 2021. Journal: Comput Math Methods Med.

**Figure 4:** Daily number of infected individuals during the Spanish COVID-19 pandemic confirmed by PCR and its trend. The figure shows the reported data (magenta line) and its trend (green line).

**Figure 5:** The Verhulst model prediction for the third wave of COVID-19 pandemic in Spain. The upper plot shows the daily number of new infections, and the lower plot the total number of infected individuals for different percentile curves (P10, P25, P50, P60, P75, P90, and P95) of the predictions.

**Figure 6:** Model parameters of the Verhulst model identified by RR-PSO. The histograms show that the maximum number of people infected in the third wave is 1.5 million and the infection rate between 0.08 and 0.1.

**Figure 7:** Daily number of infected cases (first derivative of *P*(*t*)), and the second derivative of *P*(*t*).

**Figure 8:** Spain. Percentages of the next day prediction of the daily number of people infected (daily and total), the expected deaths (*exitus*), and the urgent care units needed (UCA). Date of prediction: February, 3^rd^ 2021.

**Figure 9:** The Gompertz model prediction for the third wave of COVID-19 pandemic in Spain.

## Data Availability

Data are available upon request.

## Additional Points

*Highlights*. The Verhulst and the Gompertz models are used for the long-term prediction of new COVID-19 outbreaks. A short-term prediction model is presented based on time series analysis. Uncertainty analysis and resurgence risks are modeled. Prediction of health care needs and other correlated time series related to the COVID-19 pandemic.
